# Influence of Prehospital Emergency Care on Rescue Success Rate and Complication Rate of Senile Patients with Acute Myocardial Infarction

**DOI:** 10.1155/2022/7557288

**Published:** 2022-10-12

**Authors:** Yingchao Zhang, Lili Huang, Xuehong Zhou

**Affiliations:** Department of Emergency, Taizhou First People's Hospital, Taizhou, 318020 Zhejiang, China

## Abstract

**Objective:**

This research mainly discusses the influence of prehospital emergency care (PHEC) on the rescue success rate and complication rate of senile patients with acute myocardial infarction (AMI).

**Methods:**

We selected 200 senile AMI patients who visited between January 2019 and January 2021, and retrospectively analyzed their clinical data. According to the differences in nursing methods, the patients were assigned to control group (*n* = 90) and observation group (*n* = 110), which were treated with routine nursing and PHEC, respectively. Intergroup comparisons were made in terms of rescue success rate, nursing efficacy, clinical parameters and complication rate.

**Results:**

After investigation, the nursing efficacy was higher in the observation group compared with the control group. Additionally, the observation group was observed with statistically shorter time to thrombolysis and hospital stay, as well as evidently lower mortality and complication rates.

**Conclusion:**

The above demonstrates that PHEC can effectively improve the rescue success rate and rescue efficacy, and facilitate the recovery of senile AMI patients, with a low complication rate compared with the routine care, which plays an important role in ensuring patients' life safety and is worth popularizing clinically.

## 1. Introduction

As a serious type of coronary heart disease, acute myocardial infarction (AMI) is an important cause of cardiovascular death with an incidence that continued to rise in recent years [1]. Against the background of accelerated population aging, AMI in the elderly has become a common multiple disease in clinical cardiovascular medicine [2]. Characterized by rapid onset and fast progression, the disease is a serious threat to senile patients who are accompanied by varying degrees of decline in physical function [3]. According to the results of the World Health Organization (WHO) epidemiological study on senile AMI, the morbidity and mortality of males in all age groups (except those over 80 years old) exceeded those of females [4]. The mortality rate of AMI remains very high, despite the standardization of its diagnosis and treatment [5]. Cardiogenic shock (CGS), one of the complications of AMI, is one of the prime reasons for death in AMI patients [6]. However, at present, the clinical effect of AMI complicated with CGS leaves much to be desired, urgently demanding effective measures that can be taken to lower the incidence of complications to extend patient survival [7]. This study aims at finding a more suitable nursing method for senile AMI patients from the perspective of nursing care.

In the face of complex and rapidly developing diseases, delayed and ineffective first aid will often lead to serious adverse consequences for follow-up treatment [8]. While prehospital emergency care (PHEC) plays a vital role in providing timely and effective treatment for such patients [9]. The more accurate the judgment of the patient's condition and the faster the care given, the lower the patient's death rate between receiving the emergency task and the patient's admission [10]. At present, the PHEC model has been widely used in clinical emergency treatment of diseases such as acute cerebral infarction and acute craniocerebral trauma [11]. The report of Pendyal et al. [12] on AMI nursing process in the United States suggested that PHEC was also applicable to the first aid of AMI. Based on the conclusions of previous studies and the clinical features of senile AMI, this study attempted to introduce PHEC into the clinical treatment of elderly AMI patients.

Although there are currently many related studies on the application of PHEC in AMI, fewer of them focus on senile AMI patients. Consequently, this study mainly makes a retrospective analysis of the rescue success rate, nursing efficacy, and complications of PHEC for senile AMI patients, hoping to provide a new clinical reference for the care of senile AMI.

## 2. Data and Methods

### 2.1. Baseline Data

In this study, 200 senile patients with AMI admitted between January 2019 and January 2021 were selected and divided into an observation group (*n* = 110) and a control group (*n* = 90) according to different nursing methods. Patients in the control group received routine nursing, while those in the observation group received PHEC intervention. The control group was comprised of 51 males and 39 females who were aged 79.02 ± 10.70 years, with 26 cases presenting with inferior wall myocardial infarction, 23 cases with anterior wall myocardial infarction, 20 cases with anteroseptal myocardial infarction, and 21 cases with high lateral wall infarction. In the observation group, the male to female ratio and age range were 60 : 50 and 79.75 ± 10.11 years old, respectively, with the number of cases with inferior wall, anterior wall, anteroseptal, and high lateral wall infarction of 29, 24, 30, and 27, respectively. The two groups showed clinical comparability with similar baseline data such as sex, age, and infarction type (*P* > 0.05). This study has been approved by the hospital Ethics Committee, and all subjects and their families were aware of the study purpose and provided informed consent.

### 2.2. Eligibility Criteria

The inclusion criteria were as follows: those with a definite diagnosis of AMI; those whose age conformed to the general standard of old age division; those with no serious organ function injury; those who signed the informed consent form and actively cooperate with the treatment, with high compliance.

Patients were excluded if they met any of the following criteria: vital organ diseases, coagulation disorders, and low tolerance; severe mental diseases; treatment interruption due to various reasons; tissue infection, necrosis, etc.; patients who did not meet the inclusion criteria, were unwilling to cooperate with the study, or whose incomplete data affected the research judgment.

### 2.3. Nursing Measures

*Control Group (Routine Nursing Group)*. Patients in this group were closely monitored by medical staff for vital signs. In addition, they were given corresponding nursing care based on their actual situation and needs, as well as medication according to the doctor's advice

*Observation Group (PHEC Group)*. This group of patients received PHEC, which was conducted by a temporary first-aid team composed of experienced medical staff. After receiving the first-aid task, the first-aid team quickly understood and made a general assessment of the patient's condition. Upon arrival at the scene, the first-aid team promptly instructed the patient to lie flat to administer oxygen using a mask or nasal catheter. Furthermore, the patient's blood pressure, pulse, and other signs were detected. If the patient was found to be at risk of shock, corresponding treatment was carried out in time. On the way to the hospital, the medical staff contacted the hospital to prepare for the treatment

### 2.4. Nursing Effect Evaluation

*Marked Effectiveness*. The patient's clinical symptoms and features were significantly improved or the patient was cured without complications after nursing

Effectiveness: patients' clinical symptoms and features were obviously relieved, and the condition was basically cured after nursing, with complications in individual patients

*Ineffectiveness*. The patient died or the clinical symptoms and characteristics were not significantly improved or even worsened with complications after nursing

### 2.5. Endpoints

*Nursing Efficacy*. The nursing effect evaluation standard is described as above, and the total effective rate is the percentage of the number of (marked effectiveness + effectiveness) cases in all patients

*Rescue Success Rate*. The number of deaths and successful rescues in the two groups during care were recorded and analyzed. The percentage of successful cases in all cases was the success rate of rescue

*Clinical Parameters*. The clinical parameters such as the start time of thrombolysis and hospitalization time were recorded

*Incidence of Complications*. Complications, including arrhythmia, heart failure (HF), and CGS were observed in both groups during recovery

### 2.6. Statistical Processing

All the medical records of 200 senile AMI patients were analyzed and visualized by SPSS 21.0 (SPSS, Inc., Chicago, IL, USA) and GraphPad Prism 6 (GraphPad Software, San Diego, USA), respectively. The analysis results with *P* < 0.05 were considered statistically significant. Enumeration data (sex, age, etc.) and measurement data (average age, time from onset to rescue, etc.) were expressed by number of cases/percentage (*n*/%) and mean ± SEM, respectively. As for their statistical methods, *χ*^2^ test was used for intergroup comparisons of enumeration data, while independent samples had *t* test and paired *t* test for intergroup and intragroup comparisons of measurement data, respectively.

## 3. Results

### 3.1. Baseline Data of Senile AMI Patients

By analyzing the baseline data of 200 senile AMI patients, we found no obvious difference between the control group and the observation group in terms of sex, age, average age, time from onset to rescue, infarction type, education level, drinking history, overweight, etc., suggesting comparability (*P* > 0.05). See Table 1 for details.

### 3.2. Rescue Success Rate of Senile AMI Patients

The analysis and intergroup comparison (Table 2) of rescue success and mortality rates revealed a statistically higher rescue success rate in the observation group as compared to the control group (93.64% vs. 84.44%, *P* < 0.05).

### 3.3. Clinical Parameters of Senile AMI Patients

We recorded the time to start thrombolytic therapy and hospitalization time of the two groups to compare the effects of the two nursing methods on clinical parameters of senile AMI patients. The start time of thrombolysis and hospitalization time were found to be statistically shorter in the observation group as compared to the control group (*P* < 0.05). See Figure 1 for details.

### 3.4. Nursing Effect of Senile AMI Patients

The impacts of the two nursing methods on senile AMI patients were assessed by analyzing the nursing effects. The data identified a higher total effective rate of nursing in the observation group (92.73%) compared with the control group (80.00%), with statistical significance (*P* < 0.05, Table 3).

### 3.5. Complication Rate in Senile AMI Patients

We made an intergroup comparison regarding the incidence of complications such as arrhythmia, HF, and CGS and found that the total complication rate was statistically lower in the observation group compared with the control group (9.09% vs. 25.56%, *P* < 0.05, Table 4).

## 4. Discussion

AMI is a life-threatening condition when blood flow to the heart is suddenly blocked, causing myocardial damage or death [13]. Even though the treatment of AMI has been improved, the post-discharge mortality of patients is still very high. This is particularly true for those with complications after myocardial infarction, whose follow-up situation is even more dismal [14]. Gasior et al. [15] reported that only half of newly diagnosed HF patients managed to survive for four years, and the situation for senile patients is even less optimistic. Therefore, this study focuses on senile AMI patients and mainly analyzes the rescue success rate and complications, hoping to contribute to improving the management of senile AMI.

PHEC can provide emergency medical care for endogenous emergencies such as AMI and exogenous emergencies like burns and poisoning [16]. A previous clinical analysis shows that quite a number of AMI patients died before they arrived at the hospital [17]. On the contrary, if patients can get effective and timely prehospital first aid and are quickly transported to the hospital, the risk of death and complications will be greatly reduced [18]. This study included 200 elderly AMI patients who were divided into the control group receiving routine care and the observation group receiving PHEC according to the difference in nursing methods. The number of successfully rescued patients in the observation group was found to be significantly higher than that in the control group (93.64% vs. 84.44%), indicating that receiving PHEC can significantly improve the rescue success rate of senile AMI patients. Then, we recorded the clinical parameters of our case series. Through analysis, we found statistically shorter time to start thrombolysis and hospitalization time in the observation group compared with the control group, which suggested that the use of PHEC, an effective care model that provides timely interventions, has a positive impact on the rehabilitation process of patients. Our findings are consistent with the view that appropriate first aid, as reported by Mai et al. [19], will significantly improve patient survival chances and later treatment outcomes. In terms of nursing efficacy, a statistically higher total effective rate of nursing was determined in the observation group when compared to the control group (92.73% vs. 80.00%), demonstrating better nursing efficacy of PHEC that contributes to better nursing effects in senile AMI patients than conventional nursing. Wu et al. [20] pointed out in their report on acute stroke that the PHEC model significantly outperformed conventional emergency care in terms of nursing effect and nursing satisfaction, similar to our results.

With regard to complications, arrhythmia, HF, and CGS are the three common complications of AMI [21]. Volle et al. [22] indicated in their study that HF bore the main responsibility for morbidity and mortality in more than 10% of people over 70 years old, in addition to 10% of cases experiencing CGS immediately after the onset of AMI [23]. In our research, a statistically lower complication rate was found in the observation group as compared to the control group (9.09% vs. 25.56%), suggesting that PHEC for senile AMI patients is safer than conventional care, which is consistent with the report of Lihui and Qing [24] on the application of PHEC.

Although this paper has confirmed the beneficial effects of PHEC for senile AMI patients in increasing the rescue success rate, improving clinical indicators and nursing effects, and reducing the incidence of complications, there is still room for improvement. First of all, there is no follow-up in this study, while in fact, AMI patients have a high recurrence rate after discharge. Hence, increasing the 12-month follow-up after discharge can more intuitively determine the recovery or recurrence of patients. Second, this study is a single-center study, which is prone to information deviation. We will continue to improve the research based on the above two points in the future.

## 5. Conclusion

Collectively, PHEC for senile AMI patients is worthy of clinical promotion as it has a remarkable effect, which can not only improve the survival rate of patients but also effectively shorten their rehabilitation process and reduce complications, providing an effective nursing method for the rehabilitation of senile AMI patients.

## Figures and Tables

**Figure 1:** Clinical parameters of senile patients with acute myocardial infarction. (a) Time to start thrombolysis after nursing in the two groups. (b) Hospitalization time after nursing in the two groups. Note: ^∗∗^*P* < 0.01.

**Table 1:** Baseline data of senile patients with acute myocardial infarction [*n* (%), mean ± SEM].

Factor	*n*	Control group (*n* = 90)	Observation group (*n* = 110)	*χ* ^2^/t	*P*
Sex				0.090	0.764
Male	111	51 (56.67)	60 (54.55)		
Female	89	39 (43.33)	50 (45.45)		
Age (years old)				0.098	0.755
<80	102	47 (52.22)	55 (50.00)		
≥80	98	43 (47.78)	55 (50.00)		
Average age (years old)	200	79.02 ± 10.70	79.75 ± 10.11	0.495	0.621
Time from onset to rescue (min)	200	20.17 ± 6.62	20.90 ± 7.28	0.735	0.463
Type of infarction				0.944	0.815
Inferior wall	55	26 (28.89)	29 (26.36)		
Anterior wall	47	23 (25.56)	24 (21.82)		
Anteroseptal wall	50	20 (22.22)	30 (27.27)		
High lateral wall	48	21 (23.33)	27 (24.55)		
Education level				0.119	0.730
Technical secondary school or above	84	39 (43.33)	45 (40.91)		
Technical secondary school below	116	51 (56.67)	65 (59.09)		
Drinking history				0.232	0.630
No	77	33 (36.67)	44 (40.00)		
Yes	123	57 (63.33)	66 (60.00)		
Overweight				0.170	0.680
Yes	101	44 (48.89)	57 (51.82)		
No	99	46 (51.11)	53 (48.18)		

**Table 2:** Rescue success rate of senile patients with acute myocardial infarction [*n* (%)].

Groups	*n*	Mortality rate (%)	Rescue success rate (%)
Control group	90	14 (15.56)	76 (84.44)
Observation group	110	7 (6.36)	103 (93.64)
*χ* ^2^ value	—	—	4.450
*P* value	—	—	0.035

**Table 3:** Nursing effect of senile patients with acute myocardial infarction [*n* (%)].

Groups	*n*	Marked effectiveness	Effectiveness	Ineffectiveness	Total effective rate (%)
Control group	90	42 (46.67)	30 (33.33)	18 (20.00)	72 (80.00)
Observation group	110	74 (67.27)	28 (25.46)	8 (7.27)	102 (92.73)
*χ* ^2^ value	—	—	—	—	7.089
*P* value	—	—	—	—	0.008

**Table 4:** Complication rate in senile patients with acute myocardial infarction [*n* (%)].

Categories	Control group (*n* = 90)	Observation group (*n* = 110)	*χ* ^2^ value	*P* value
Arrhythmia	12 (13.33)	5 (4.55)	—	—
Heart failure	6 (6.67)	3 (2.72)	—	—
Cardiogenic shock	5 (5.56)	2 (1.82)	—	—
Total incidence	23 (25.56)	10 (9.09)	9.740	0.002

## Data Availability

The labeled dataset used to support the findings of this study are available from the corresponding author upon request.

## References

[1] Cui C. Y., Zhou M. G., Cheng L. C. (2021). Admission hyperglycemia as an independent predictor of long-term prognosis in acute myocardial infarction patients without diabetes: a retrospective study. *Journal of Diabetes Investigation*.

[2] Van de Werf F. (2018). Reperfusion treatment in acute myocardial infarction in elderly patients. *Kardiologia Polska*.

[3] Kapur N. K., Thayer K. L., Zweck E. (2020). Cardiogenic shock in the setting of acute myocardial infarction. *Methodist DeBakey Cardiovascular Journal*.

[4] Tukish O. V., Okrugin S. A., Yunusova E. Y., Efimova E. V., Garganeeva A. A. (2016). Acute myocardial infarction in elderly and senile patients: epidemiology study according to the who program “registry of acute myocardial infarction”. *Advances in Gerontology*.

[5] Li J., Li X., Wang Q. (2015). ST-segment elevation myocardial infarction in china from 2001 to 2011 (the China peace-retrospective acute myocardial infarction study): a retrospective analysis of hospital data. *Lancet*.

[6] Tokunaga C., Iguchi A., Nakajima H. (2022). Surgical outcomes of bridge-to-bridge therapy with extracorporeal left ventricular assist device for acute myocardial infarction in cardiogenic shock. *BMC Cardiovascular Disorders*.

[7] Nishi T., Ishii M., Tsujita K. (2022). Outcomes of venoarterial extracorporeal membrane oxygenation plus intra-aortic balloon pumping for treatment of acute myocardial infarction complicated by cardiogenic shock. *Journal of the American Heart Association*.

[8] Wang L., Wu R. (2021). Clinical effectiveness of pre-hospital and in-hospital optimized emergency care procedures for patients with acute craniocerebral trauma. *Frontiers in Surgery*.

[9] Hsia R. Y., Huang D., Mann N. C. (2018). A US national study of the association between income and ambulance response time in cardiac arrest. *JAMA Network Open*.

[10] Dehghan-Nayeri N., Nouri-Sari H., Bahramnezhad F., Hajibabaee F., Senmar M. (2021). Barriers and facilitators to cardiopulmonary resuscitation within pre-hospital emergency medical services: a qualitative study. *BMC Emergency Medicine*.

[11] Moreno-Carrillo A., Arenas L. M. A., Fonseca J. A., Caicedo C. A., Tovar S. V., Munoz-Velandia O. M. (2019). Application of queuing theory to optimize the triage process in a tertiary emergency care ("ER") department. *Journal of Emergencies, Trauma, and Shock*.

[12] Pendyal A., Rothenberg C., Scofi J. E. (2020). National trends in emergency department care processes for acute myocardial infarction in the United States, 2005 to 2015. *Journal of the American Heart Association*.

[13] Lee J., Lee S., Street W. N., Polgreen L. A. (2022). Machine learning approaches to predict the 1-year-after-initial-AMI survival of elderly patients. *BMC Medical Informatics and Decision Making*.

[14] Chen D. Y., Li C. Y., Hsieh M. J. (2019). Predictors of subsequent myocardial infarction, stroke, and death in stable post-myocardial infarction patients: a nationwide cohort study. *European Heart Journal Acute Cardiovascular Care*.

[15] Gasior M., Wita K., Buszman P. (2022). Managed care after acute myocardial infarction (MC-AMI) improves prognosis in AMI survivors with pre-existing heart failure: a propensity score matching analysis of Polish nationwide program of comprehensive post-MI care. *Kardiologia Polska (Polish Heart Journal)*.

[16] Wake K., Noguchi T., Hishinuma H. (2022). Characteristics of patients who received helicopter emergency medical services in Japan from 2012 to 2019: a retrospective analysis of data from Tochigi prefecture. *Scandinavian Journal of Trauma, Resuscitation and Emergency Medicine*.

[17] Rosell-Ortiz F., Mellado-Vergel F. J., Fernandez-Valle P. (2015). Initial complications and factors related to prehospital mortality in acute myocardial infarction with ST segment elevation. *Emergency Medicine Journal*.

[18] Najafi H., Bahramali E., Bijani M., Dehghan A., Amirkhani M., Balaghi Inaloo M. (2022). Comparison of the outcomes of ems vs. non-EMS transport of patients with ST-segment elevation myocardial infarction (STEMI) in southern Iran: a population-based study. *BMC Emergency Medicine*.

[19] Mai H. T., Vu H. M., Ngo T. T. (2020). The status of first aid and its associations with health outcomes among patients with traffic accidents in urban areas of Vietnam. *International Journal of Environmental Research and Public Health*.

[20] Wu Y., Yang Y., Guo X. (2022). Effect of pre-hospital early intervention combined with an in-hospital emergency model in the emergency care of patients with acute stroke. *American Journal of Translational Research*.

[21] Petersen L. T., Riddersholm S., Andersen D. C. (2021). Temporal trends in patient characteristics, presumed causes, and outcomes following cardiogenic shock between 2005 and 2017: a Danish registry-based cohort study. *European Heart Journal Acute Cardiovascular Care*.

[22] Volle K., Delmas C., Rollin A. (2021). Successful reversal of severe tachycardia-induced cardiomyopathy with cardiogenic shock by urgent rhythm or rate control: only rhythm and rate matter. *Journal of Clinical Medicine*.

[23] Samsky M. D., Morrow D. A., Proudfoot A. G., Hochman J. S., Thiele H., Rao S. V. (2021). Cardiogenic shock after acute myocardial infarction: a review. *JAMA*.

[24] Lihui L., Qing Y. (2021). Optimizing the prehospital-hospital emergency care path application value in emergency treatment of patients with cerebral hemorrhage. *Journal of Healthcare Engineering*.

